The article "Mothers’ and Fathers’ Science-Related Talk With Daughters and Sons While Reading Life and Physical Science Books" was published in 2022. Journal: Front Psychol.

# Mothers’ and Fathers’ Science-Related Talk With Daughters and Sons While Reading Life and Physical Science Books

**DOI:** 10.3389/fpsyg.2021.813572

**Published:** 2022-02-14

**Authors:** Tess A. Shirefley, Campbell Leaper

**Affiliations:** Department of Psychology, University of California, Santa Cruz, Santa Cruz, CA, United States

**Keywords:** gender differences, mother-child communication, father-child communication, reading, science education

## Abstract

**Introduction:**

In prior studies conducted in the United States, parents’ gender-differentiated encouragement of science predicted children’s later science motivation. Most of this research has focused on older children or teens and only looked at the impact of mothers. However, accumulating evidence suggests that gender-differentiated encouragement of science interest may begin in early childhood. Moreover, fathers may be more likely than mothers to treat sons and daughters differently in science-learning contexts.

**Methods:**

We examined 50 United States families with both a mother and a father (82% White; 98% with at least some college education) and either a daughter or a son (48–83 months; *M* = 62, *SD* = 9). On separate visits, each parent reads two books with their child. One was about life science and the other was about physical science. We coded parents’ science-related talk during these interactions.

**Results and Conclusion:**

In contrast to our predictions, parents used higher proportions of science talk with daughters than sons, including higher average rates of overall science talk and specific types of science talk (e.g., science explanations, science-related personal connections, and science-learning talk). Moreover, most of the child gender effects occurred while reading the physical science books. Book topic and parent gender moderated some additional patterns. Book reading is discussed as a potential context for mitigating socialization experiences that traditionally disfavor girls’ interest in physical science.

## Introduction

Even though women and men demonstrate comparable levels of participation in the life science workforce in the United States, women remain underrepresented in physical science domains (National Science Foundation, 2021). As documented in earlier reports, interest in physical science more likely increased from middle childhood to adolescence among boys than girls; in contrast, interest in life science remained comparable for girls and boys during this period (e.g., Baram-Tsabari and Yarden, 2008). The development of average gender differences in motivation and achievement is attributed to a combination of individual, interpersonal, and cultural factors (Cheryan et al., 2017; Eccles and Wigfield, 2020). Among them, researchers have highlighted the potential impact of parents’ gender-differentiated socialization on children’s developing interests and ability beliefs (Eccles and Wigfield, 2020). We built on prior research in three ways. First, previous research on parents’ gender-differentiated socialization of their children’s science learning and interest has focused on middle childhood and adolescence. Hence, we explored whether the gender-differentiated patterns might be detected in a younger age group of children between 4 and 7 years of age. Second, previous research studies looked primarily at mothers without considering parent gender as a potential moderator. We examined children’s book reading separately with their mothers and fathers. Finally, scant research has separately examined physical science and life science when considering parents’ gender-differentiated treatment. Hence, we observed parents reading separate science books on life science and physical science with their children.

The article "Mothers’ and Fathers’ Science-Related Talk With Daughters and Sons While Reading Life and Physical Science Books" was published in 2022. Journal: Front Psychol.

### Parents’ Gender-Differentiated Socialization of Children’s Science Interest

Longitudinal studies established how parents’ gender-differentiated beliefs about their children’s science, technology, engineering, and mathematics (STEM)-related interests or abilities predicted later changes in children’s motivational beliefs and achievement (e.g., Simpkins et al., 2015). However, if parents’ gender-stereotyped expectations matter, then how are they manifested in their interactions with their children at young ages? According to ecological and social cognitive theories of development (Bussey and Bandura, 1999; Bronfenbrenner, 2005), this can occur when parents provide different opportunities for learning to children based on their gender. For example, this was indicated by Tenenbaum and Leaper (2003) in their observations of parents with their 10-year-old daughter or son while engaging in assigned science activities. On average, fathers (but not mothers) used more science-related talk (e.g., explanations, scientific vocabulary) with their sons than daughters during a physical science task. But other studies suggest that this kind of gender-differentiated treatment may occur at much younger ages. In at least three studies, parents of preschool-age children were observed talking more about science with their sons than daughters. These effects were observed at a science museum (Crowley et al., 2001) while playing with a physics toy at home (Tenenbaum et al., 2005) and reading a science-related book (Shirefley et al., 2020). Although the evidence is limited, two studies suggest that gender-related variations might occur with some types of science talk more than others (Tenenbaum et al., 2005; Shirefley et al., 2020).

The article "Mothers’ and Fathers’ Science-Related Talk With Daughters and Sons While Reading Life and Physical Science Books" was published in 2022. Journal: Front Psychol.

### Shared Book Reading as a Context for Investigating Parents’ Talk With Young Children

Shared book reading is a common context in many families where informal learning for young children occurs with their parents (Scholastic Inc, 2016). More specifically, researchers have highlighted how parents’ book reading with preschool-age children was a means for discussing and learning complex science concepts (e.g., Kelemen et al., 2014; Shirefley et al., 2020) and imparting lessons about gender roles (e.g., Friedman et al., 2007; Endendijk et al., 2014). However, no prior work has considered how conversations during shared reading may vary with the type of science book (life vs. physical) or with both mothers and fathers.

### Comparing Fathers’ and Mothers’ Science Talk With Children

When considering parents’ gender as a moderator of science talk, two patterns have been previously identified. First, average differences between mothers’ and fathers’ behavior with their children may occur (refer to Leaper, 2015 for review). Some studies have found that mothers were more verbal than fathers when interacting with children (refer to Leaper et al., 1998 for a meta-analysis). Only a few studies have compared mothers’ and fathers’ verbal behavior specifically during shared reading with their young children. Their results have been mixed. Two studies observed greater talking or more teaching-related comments among mothers than fathers (Conner et al., 1997; Schwartz, 2004). One study noted more talking among fathers than mothers (Anderson et al., 2004). In addition, another investigation found negligible differences between mothers’ and fathers’ teaching-related speech during shared reading (Blake et al., 2006). None of these studies, however, observed the shared reading of books focused on science topics.

A second pattern regarding parent gender differences indicated in the research literature is for fathers to be more likely than mothers to treat daughters and sons differently (refer to Leaper, 2015). Regarding science-related talk with young children, one study observed that both mothers and fathers used more science talk with boys than girls at a science museum, but the trend was stronger among fathers (Crowley et al., 2001). We do not know whether similar patterns would be seen while reading science books.

In addition, research with older children suggests that differences between fathers and mothers in gender-differentiated encouragement of science may partly depend on the type of science. Two studies looked at mothers’ and fathers’ hands-on involvement with elementary-school-age children in both life science and physical science tasks. In the first study, fathers used more science-teaching talk with sons than daughters but only during the physical science task; conversely, mothers did not differ with daughters and sons in either task (Tenenbaum and Leaper, 2003). In the second study, researchers surveyed parents based on the kinds of science problems they solved with their children (Short-Meyerson et al., 2016). Mothers favored more life science tasks, whereas fathers preferred more physical science tasks. From these studies, there is evidence to suggest that average differences in mothers’ and fathers’ behavior may occur when reading science books to their young children. Accordingly, we took into account the parent gender, the child gender, and the type of science book being read.

The article "Mothers’ and Fathers’ Science-Related Talk With Daughters and Sons While Reading Life and Physical Science Books" was published in 2022. Journal: Front Psychol.

### Current Study

To build on earlier research investigating parents’ science-related talk with children, we observed parents with their 4–7-year-old children while reading physical and life science books in their homes. We chose book reading as it is a common shared activity among many parents and their young children, and it is an activity that is easily arranged in families’ homes. We tested for variations in parents’ science-related talk by child gender, parent gender, and the type of science book. Our hypotheses were as follows: first, we expected that parents would use a greater proportion of science-related talk with their sons than daughters. Second, we predicted that parents’ gender-differentiated science talk would be more likely for fathers than mothers. Finally, we hypothesized that these effects would be stronger when reading the physical science book. When conducting our analyses, we looked at parents’ overall science talk. In addition, we examined specific forms of science talk to explore whether some might be related to gender-related variations more than others. Among the few studies that examined parents’ science talk, none of them considered whether gender-differentiated treatment was more likely for some forms of science talk than others.

## Methods

### Participants

Participants were recruited in northern California through social media posts, local community spaces, and preschools. This study focuses on families in our sample with heterosexual parents in which both the mother and the father were able to participate, which initially comprised 55 families. Of these families, five were removed due to technical difficulties (*n* = 2) or child non-compliance with the tasks (*n* = 3). Our analyses are based on 50 families with a participating daughter or son (*n* = 25 each) between 4 and 7 years of age (*M* = 62 months, *SD* = 9.5). The average age of daughters and sons did not significantly differ. For mothers, 82% self-identified as White and 88% had attained at least a bachelor’s degree. For fathers, 82% self-identified as White and 74% had attained at least a bachelor’s degree (refer to Table 1 for more detail). Parent-child dyads were asked to read and discuss the books as it was most natural to them (*n* = 48 exclusively in English, *n* = 1 in English and Spanish, and *n* = 1 in English and German).

The article "Mothers’ and Fathers’ Science-Related Talk With Daughters and Sons While Reading Life and Physical Science Books" was published in 2022. Journal: Front Psychol.

**TABLE 1:** Demographic backgrounds of mothers and fathers.

Variable	Mothers	Fathers
**Ethnicity**		
*White*	41	41
*Latinx*	5	6
*Asian/Pacific Islander*	1	2
*Black*	1	0
*Multi/Other*	2	1
**Education level**		
*High school diploma*	1	1
*Some college/Associate’s*	5	12
*College bachelors*	19	20
*Masters/Doctorate/Medical*	25	17

## Materials and Procedure

### Science Books

We selected four science books from the *Let’s Read-and-Find-Out Science* series by HarperCollins written for preschool-aged children. All books were in English. Two different books focused on physical science [*What Is The World Made Of?* (about solids, liquids, gasses) and *Light Is All Around Us* (how light brightens the world)] and two books were on life science [*From Seed to Pumpkin* (process of a pumpkin growing) and *From Caterpillar To Butterfly* (transformation from caterpillar to butterfly)]. We edited the four books to balance the proportion of science-related content across books. Each book was about 13 pages with approximately 30% of the text containing science words.

After obtaining signed consent, parent-child dyads were video-recorded while reading one life science book and one physical science book (with different versions provided to mothers and fathers). No time limit was imposed. The order of books and the versions of each book type were counterbalanced across parent gender and child gender. We attempted to counterbalance the order of visits with mothers and fathers; however, several fathers would not participate in the study unless mothers participated first. Mothers were visited first in 17 of 25 families with daughters and 16 of 25 families with sons. Home visits were conducted 1–2 weeks apart.

After parents completed the reading of the science books, they completed a brief survey assessing their attitudes and beliefs about science. Among these questions, two items assessed their beliefs about their child’s science ability and interest (from Tenenbaum and Leaper, 2003): “My child finds science (0 = *very boring* to 7 = *very interesting*)” and “My child finds science…(0 = *very hard* to 7 = *very easy*).” Also, we asked “How often do you read a storybook to your child?” (0 = *never*, 1 = *a few times per year*, 2 = *about once per month*, 3 = *about once per week*, and 4 = *almost every day*).

The article "Mothers’ and Fathers’ Science-Related Talk With Daughters and Sons While Reading Life and Physical Science Books" was published in 2022. Journal: Front Psychol.

### Coding

We first transcribed parent-child video recordings using Datavyu. We parsed parent-child talk into utterances representing individual thought units. Parent and child utterances were coded into 16 coding categories, which included five science-related codes (based on Shirefley et al., 2020). Five research assistants coded 20% of the dataset to assess intercoder reliability. After achieving reliability and discussing differences, each coder coded 20% of the remaining samples. The five types of the science-related talk were as follows: *scientific explanations*, *science labels*, *scientific personal connections*, *scientific story inferences*, and *scientific-learning talk* (refer to Table 2 for definitions and Table 3 for descriptive statistics). Based on the guidelines developed by Landis and Koch (1977), the intercoder agreement for each code was acceptable (refer to Table 2).

**TABLE 2:** Science talk codes: descriptions and intercoder reliability.

Measure	Definition	Percent agreement	Kappa coefficient	Evaluation^1^
Scientific explanations	Generic facts vocabulary and explanations about a phenomenon specifically related to the scientific material (e.g., “Roots suck up water like a straw”).	88	0.66	Substantial
Science labels	The naming of a specific part of an image within the book (e.g., “Those are called pupa”).	95	0.65	Substantial
Scientific personal connections	Relating the scientific material of the book to a child/parent/family’s prior experience (e.g., “Remember when we made Play-Doh and at first it was really liquidy but then we added more starch to make it solid?”).	95	0.72	Substantial
Scientific story inferences	Anticipating the next step in the story (taking information not visible on the page of the book to then infer understanding (e.g., “There was a lot of rain, I wonder what will happen to the pumpkin seeds”).	99	0.37	Fair
Scientific-learning talk	A reference to new scientific knowledge gained or the opportunity for parent or child to check in with each other about their understanding of information (e.g., “Did you know the sun was that hot?!”).	96	0.42	Moderate

*^1^Source: Landis and Koch (1977).*

*Story inferences occurred infrequently (refer to Table 3), which likely accounts for the relatively low intercoder agreement.*

**TABLE 3:** Mean frequencies and proportions for science-related talk variables of parents.

	Frequencies		Proportions	
	Life science	Physical science	Life science	Physical science
	*M* (*SD*)	*M* (*SD*)	*M* (*SD*)	*M* (*SD*)
Total talk	50.8 (25.5)	53.3 (36.7)	N/A	N/A
Overall science talk	30.8 (17.8)	37.8 (24.4)	0.60 (0.13)	0.59 (0.14)
Scientific explanations or vocabulary	13.0 (10.5)	22.6 (18.1)	0.24 (0.12)	0.34 (0.14)
Science labels	5.7 (4.3)	3.7 (4.4)	0.12 (0.09)	0.06 (0.06)
Scientific personal connections	6.7 (5.5)	6.7 (6.2)	0.14 (0.09)	0.11 (0.08)
Scientific story inferences	0.8 (2.1)	0.3 (0.6)	0.01 (0.03)	0.004 (0.01)
Scientific-learning talk	4.5 (3.8)	4.9 (4.1)	0.09 (0.05)	0.08 (0.05)

*N/A, not applicable.*

The article "Mothers’ and Fathers’ Science-Related Talk With Daughters and Sons While Reading Life and Physical Science Books" was published in 2022. Journal: Front Psychol.

*The total talk reflects all utterances excluding reading text from the book. Proportion scores reflect the proportions of each science talk variable in relation to parents’ total utterances (excluding reading text from book).*

## Results

### Statistical Design

Children were observed on separate occasions with their mother and father, and each parent reads two types of science books. Because members of dyads are not independent, we utilized linear mixed models to conduct our analyses (Kenny et al., 2006). Child gender was a between-group factor, whereas parent gender and book type were nested factors. The mixed linear model is only able to examine one criterion variable at a time. Accordingly, we ran six models with parents’ overall science talk and the five specific types of science talk. To control for variations across parents in the time spent talking about the book, we calculated each type of science talk as a proportion of total utterances (excluding reading text from the book).

### Preliminary Analyses

We conducted preliminary analyses to test for gender-related variations in a few factors that might influence parents’ gender-differentiated talk. First, we did not find significant differences in parents’ views of daughters’ and sons’ science ability or interest, although mothers were more likely than fathers to rate their children as finding science easy (*p* = 0.032). Second, we did not find differences in parents’ reported reading to daughters vs. sons. Indeed, 94% of mothers and 90% of fathers reported reading to their children “almost every day.” Finally, we did not find differences between daughters’ and sons’ total talk and science-related talk with either science book, although children used proportionally more science talk with the life science book than the physical science book (*p* < 0.001).

### Testing Hypotheses

In summarizing the results below, only significant effects from the models are noted (refer to Table 4 for more information). With any significant pairwise comparisons tests, Cohen’s *d* indices of effect size are reported. Effect sizes are negligible when *d* < 0.2 (or η^2^ < 0.01), small when *d* = 0.2 (or η^2^ = 0.01), moderate when *d* = 0.5 (or η^2^ = 0.06), and large when *d* = 0.8 (or η^2^ = 0.14) or greater (Cohen, 1988).

The article "Mothers’ and Fathers’ Science-Related Talk With Daughters and Sons While Reading Life and Physical Science Books" was published in 2022. Journal: Front Psychol.

**TABLE 4:** Summary of results from linear mixed models.

	Overall	Explanations	Labels	Connections	Inferences	Learning
	*F*_(1,46)_	*F*_(1,47)_	*F*_(1,48)_	*F*_(1,48)_	*F*_(1,47)_	*F*_(1,47)_
Child gender (CG)	4.70*	4.14*	0.07	0.27	0.17	8.98**
Parent gender (PG)	1.46	1.64	0.63	0.64	2.42	0.65
Book type (BT)	0.38	63.57***	44.75***	9.62**	11.92***	2.14
CG × BT	5.24*	1.03	0.01	7.33*	0.29	7.15**
PG × BT	0.32	1.15	0.05	2.07	6.93*	1.25
CG × PG	0.13	0.02	0.01	1.61	0.16	8.36**
CG × PG × BT	0.33	0.43	0.03	0.33	0.04	0.18

*p < 0.05, **p < 0.01, and ***p < 0.001.

### The Proportion of Overall Science Talk

The main effect of child gender occurred whereby parents used more overall science talk with daughters (*M* = 0.62, *SD* = 0.12) than sons (*M* = 0.57, *SD* = 0.15), *F*_(1,46)_ = 4.70, *p* = 0.035, η^2^_*partial*_ = 0.09, *d* = 0.37. This main effect was subsumed by a Science Topic × Child Gender interaction, *F*_(1,46)_ = 4.50, *p* = 0.040, η^2^_*partial*_ = 0.09. Follow-up pairwise comparisons revealed that parents reading the physical science book used a higher average proportion of overall science talk with daughters (*M* = 0.64, *SD* = 0.13) than sons (*M* = 0.55, *SD* = 0.14), *p* = 0.003, *d* = 0.67. Parents did not significantly differ in their overall science talk with daughters (*M* = 0.62, *SD* = 0.11) and sons (*M* = 0.59, *SD* = 0.16) when reading the life science book.

### The Proportion of Science Explanations

A significant main effect of child gender indicated that parents were more likely to use science explanations with daughters (*M* = 0.31, *SD* = 0.15) than sons (*M* = 0.26, *SD* = 0.14), *F*_(1,47)_ = 4.60, *p* = 0.037, η^2^_*partial*_ = 0.09. Also, a significant main effect of science topic revealed that parents were more likely to use science explanations when reading the physical science book (*M* = 0.34, *SD* = 0.15) than the life science book (*M* = 0.22, *SD* = 0.12), *F*_(1,47)_ = 63.57, *p* = 0.003, η^2^_*partial*_ = 0.18.

### The Proportion of Science Labeling

A main effect of science topic indicated that parents used proportionally more scientific labels on average when reading the life science book (*M* = 0.12, *SD* = 0.09) than the physical science book (*M* = 0.06, *SD* = 0.06), *F*_(1, 48)_ = 44.75, *p* < 0.001, η^2^_*partial*_ = 0.10.

### The Proportion of Science Personal Connections

Based on the main effect of science books, parents were more likely to make science-related personal connections when reading the life science book (*M* = 0.14, *SD* = 0.09) than the physical science book (*M* = 0.10, *SD* = 0.08), *F*_(1,48)_ = 9.62, *p* = 0.001, η^2^_*partial*_ = 0.20. In addition, there was a significant Science Topic × Child Gender interaction, *F*_(1,48)_ = 6.10, *p* = 0.017, η^2^_*partial*_ = 0.12. Follow-up pairwise comparison tests revealed child gender differences based on the science topic. When reading the physical science book, parents made more science-related personal connections with daughters (*M* = 0.13, *SD* = 0.09) than sons (*M* = 0.08, *SD* = 0.05), *p* = 0.04, *d* = 0.69. When reading the life science book, parents did not significantly differ in their use of scientific personal connections with daughters (*M* = 0.13, *SD* = 0.08) and sons (*M* = 0.15, *SD* = 0.11).

The article "Mothers’ and Fathers’ Science-Related Talk With Daughters and Sons While Reading Life and Physical Science Books" was published in 2022. Journal: Front Psychol.

### The Proportion of Science Inferences

The main effect of science topic revealed that parents used significantly more science inferences when reading the life science book (*M* = 0.01, *SD* = 0.03) than the physical science book (*M* = 0.00, *SD* = 0.01), *F*_(1,47)_ = 11.92, *p* = 0.003, η^2^_*partial*_ = 0.17. A significant Parent Gender × Science Topic interaction [*F*_(1,47)_ = 6.9, *p* = 0.011, η^2^_*partial*_ = 0.13] indicated a significant parent gender difference depending on science topic. On average, fathers (*M* = 0.02, *SD* = 0.04) were more likely than mothers (*M* = 0.01, *SD* = 0.02) to use science inferences when reading the life science book, *p* = 0.012, *d* = 0.47; but mothers (*M* = 0.01, *SD* = 0.01) and fathers (*M* = 0.00, *SD* = 0.06) did not significantly differ when reading the physical science book.

### The Proportion of Science-Learning Talk

A significant main effect of child gender showed that parents generally used more science-learning talk with daughters than sons, *F*_(1,47)_ = 10.5, *p* = 0.002, η^2^_*partial*_ = 0.19. However, this effect was subsumed into two interaction effects. First, there was a Child Gender × Parent Gender interaction, *F*_(1,47)_ = 9.6, *p* = 0.003, η^2^_*partial*_ = 0.17. Follow-up pairwise comparison tests revealed that mothers used proportionally more science-learning talk with daughters (*M* = 0.11, *SD* = 0.06) than sons (*M* = 0.05, *SD* = 0.04), *p* < 0.001, *d* = 1.08. There was no significant difference in fathers’ science-learning talk with daughters (*M* = 0.08, *SD* = 0.05) and sons (*M* = 0.08, *SD* = 0.05). Also, a significant Child Gender × Science Topic interaction occurred, *F*_(1,47)_ = 9.5, *p* = 0.003, η^2^_*partial*_ = 0.17. On average, while reading the life science book, parents used a higher proportion of science-learning talk with daughters (*M* = 0.11, *SD* = 0.06) than sons (*M* = 0.06, *SD* = 0.05), *p* < 0.001, *d* = 0.91. There were no significant differences in science-learning talk used between daughters (*M* = 0.08, *SD* = 0.06) and sons (*M* = 0.07, *SD* = 0.05) when reading the physical science book.

The article "Mothers’ and Fathers’ Science-Related Talk With Daughters and Sons While Reading Life and Physical Science Books" was published in 2022. Journal: Front Psychol.

## Discussion

Our findings revealed patterns of gender differentiation in the science talk of mothers and fathers when reading physical and life science books to their sons or daughters. In contrast to our hypothesis, parents used a higher proportion of several forms of science talk with daughters compared to sons. Moreover, the magnitudes of these average differences were moderate-to-large in size. The science topic moderated some of these differences and parent gender moderated child gender differences although not always in an expected manner. Also, gender-related differences occurred across various types of science talk. As discussed below, the results suggested that science book reading with young children may be a context in some families in which parents may especially engage girls in science learning.

To the best of our knowledge, only three prior studies examined gender differences in parents’ science talk with preschool- and early elementary-aged children. In these investigations, parents were more likely to use science explanations with boys than girls at a science museum (Crowley et al., 2001) while playing with a science activity at home (Tenenbaum et al., 2005) or reading a science-related book (Shirefley et al., 2020). We observed the opposite pattern whereby parents generally used more scientific explanations and overall science talk with their daughters than sons across both books. In addition, mothers (but not fathers) used more science-learning talk with daughters than sons across both books.

The science topic moderated some additional effects. When reading the physical science book, parents used proportionally more overall science talk and made more science-related personal connections with their daughters than sons. Given the gender gap in motivation and achievement in the physical sciences observed during adolescence, i.e., when boys have often participated in the physical sciences than girls (refer to Cheryan et al., 2017), this pattern was surprising.

Our sample comprised mothers and fathers who generally were highly educated and active readers with their children. Perhaps these parents made concerted efforts to counteract cultural stereotypes about gender and science (e.g., physical sciences being stereotypically masculine). In doing so, they may have sought to engage their daughters especially in the science topic that was most counter-stereotypical. Mothers, in particular, may have been focused on this goal, as we found mothers but not fathers used more science-learning talk with daughters than sons. Families in our study also lived near many scientific/technology industries and in communities where issues of gender and STEM are often highlighted in local and national media. In one pertinent study, researchers discovered that girls’ enrollment in high school physics courses was higher in communities where women were employed in nearby STEM occupations (Riegle-Crumb and Moore, 2014). An analogous effect may be occurring with our sample. Of course, this interpretation is speculative and requires testing in future research.

The article "Mothers’ and Fathers’ Science-Related Talk With Daughters and Sons While Reading Life and Physical Science Books" was published in 2022. Journal: Front Psychol.

Another potential explanation for parents’ greater average science talk with daughters than sons is that parents were responding to subtle gender differences in children’s behavior (Bell, 1968). On average, girls tend to do somewhat better in reading (Robinson and Theule Lubienski, 2011) and to be more talkative during early childhood (Leaper and Smith, 2004). Although we did not find average gender differences in children’s overall science talk, perhaps girls were more likely receptive to shared book reading and parents found it easier to engage them in science talk. If so, why was parents’ science talk more likely among girls (vs. boys) specifically while reading the physical science book? Perhaps engaging the child’s interest was more challenging while discussing the more abstract physical science books than the more concrete life science books. Once again, these are speculations that need testing.

In contrast to several prior studies indicating gender-differentiated socialization was more likely among fathers than mothers (refer to Leaper, 2015 for review), we did not observe this in the results. We did observe that fathers were more likely than mothers to make scientific inferences while reading the life science book. Perhaps fathers were generally more comfortable to make these more abstract and cognitively demanding forms of talk (e.g., Tenenbaum and Leaper, 1998). Fathers could also be less familiar than mothers with their children’s cognitive abilities, which might lead to using more complex talk. Given that the science inference code was infrequent, these interpretations should be viewed cautiously.

One notable limitation of our study is that our sample was comprised of parents from highly educated backgrounds who also regularly read to their children. Prior study has noted that parents’ shared book reading is positively correlated with their education (e.g., Yarosz and Barnett, 2001). Therefore, shared book reading is not a common activity in all families. Another limitation was that the parents in our study were predominantly from White European-heritage backgrounds. Other research suggests that gender-differentiated talk in reading and other learning tasks may vary across different ethnic or cultural groups (e.g., Shirefley et al., 2020).

The article "Mothers’ and Fathers’ Science-Related Talk With Daughters and Sons While Reading Life and Physical Science Books" was published in 2022. Journal: Front Psychol.

## Conclusion

Our findings pose new research questions regarding parents’ gender-differentiated encouragement of children’s science interest, confidence, and achievement. In contrast to prior studies, we discovered that parents used the more scientific talk with their daughters than sons. This was especially likely with the physical science book. Although more research is needed to replicate and better understand the results, one possibility is that shared book reading could be a learning context conducive for promoting science interest in many girls. To test this premise, short-term longitudinal studies could examine whether this type of book reading in early childhood is related to an increase in girls’ interest in physical science. Moreover, similar benefits may accrue to boys and thereby help all children’s developing interest in science.

## Data Availability Statement

The raw data supporting the conclusions of this article will be made available by the authors, without undue reservation.

## Ethics Statement

The studies involving human participants were reviewed and approved by the University of California, Santa Cruz Institutional Review Board. Written informed consent to participate in this study was provided by the adult participants and the legal guardian of the minor participants.

## Author Contributions

TS was largely responsible for data collection, coding, and the data analyses. Both authors worked on writing the report and developed the research questions and methodology.

## Conflict of Interest

The authors declare that the research was conducted in the absence of any commercial or financial relationships that could be construed as a potential conflict of interest.

## Publisher’s Note

All claims expressed in this article are solely those of the authors and do not necessarily represent those of their affiliated organizations, or those of the publisher, the editors and the reviewers. Any product that may be evaluated in this article, or claim that may be made by its manufacturer, is not guaranteed or endorsed by the publisher.
